The article "Study of TCM Syndrome Identification Modes for Patients with Type 2 Diabetes Mellitus Based on Data Mining" was published in 2021. Journal: Evid Based Complement Alternat Med.

# Study of TCM Syndrome Identification Modes for Patients with Type 2 Diabetes Mellitus Based on Data Mining

**DOI:** 10.1155/2021/5528550

**Published:** 2021-09-06

**Authors:** Tieniu Zhao, Xiaonan Yang, Ruixin Wan, Lihui Yan, Rongrong Yang, Yuanyuan Guan, Dongjun Wang, Huijun Wang, Hongwu Wang

**Affiliations:** ^1^School of Health Science and Engineering, Tianjin University of Traditional Chinese Medicine, Tianjin 301617, China; ^2^Department of Internal Medicine, Tianjin Hongqiao District Hospital of Traditional Chinese Medicine, Tianjin 300131, China; ^3^Technology and Culture Exchange Center, China Soong Ching Ling Youth Science, Beijing 100080, China; ^4^NHC Key Laboratoryo f Hormones and Development, Tianjin Key Laboratory of Metabolic Diseases, Chu Hsien-I Memorial Hospital & Tianjin Institute of Endocrinology, Tianjin Medical University, Tianjin 300134, China; ^5^Department of Public Health, School of Health Science and Engineering, Tianjin University of Traditional Chinese Medicine, Tianjin 301617, China; ^6^Graduate School, Tianjin University of Traditional Chinese Medicine, Tianjin 301617, China; ^7^Department of Typhoid, School of Chinese Medicine, Tianjin University of Traditional Chinese Medicine, Tianjin 301617, China

## Abstract

**Objective:**

To establish the diagnosis model for syndromes of type 2 diabetes mellitus (T2-DM) and explore symptoms, the pulse and tongue signs, and laboratory indexes related to syndromes of T2-DM.

**Methods:**

A syndromatologic and laboratory investigation was conducted in 554 T2-DM patients with 58 symptoms, 14 tongue signs, 6 pulse signs, and 12 laboratory indexes. The clinical data on the syndrome were collected and analyzed by using logistic regression analysis, decision tree, and *K*-nearest neighbor to establish a diagnostic model for effectively distinguishing the typical syndromes in T2-DM patients.

**Results:**

The most typical syndromes revealed in T2-DM were stomach heat flourishing (SHF) syndrome (261 patients, accounting for 47.1%) and Qi-Yin deficiency (QYD) syndrome (293 patients, 52.9%). According to the clinical data of the patients with these two syndromes, variables including 6 symptoms and signs, 2 pulse signs, 1 tongue sign, and 2 laboratory indicators were introduced into the logistic regression model. All of them were statistically significant. Then, a diagnostic model constructed by QUEST and CHAID algorithms of the decision tree for identifying the two syndromes was proved to have an accurate diagnostic rate of 85.2%. It was found that the following sign and symptoms were effective to differentiate these two syndromes: odor in the mouth, polyphagia, vulnerability to starvation, burning sensation in the stomach, fatigue, limb weakness, slippery and replete pulse, weak pulse, pink tongue, oral glucose tolerance test, and hemoglobin A1C. A classification model constructed by the *K*-nearest neighbor method to identify the two syndromes showed an accurate diagnostic rate of 88.3%. Three major statistically significant predictors included in the model were slippery and replete pulse, polyphagia, and weak pulse (*P* < 0.05).

**Conclusion:**

A model for distinguishing the two typical syndromes (SHF syndrome and QYD syndrome) in T2-DM patients was effectively established. This model could help to provide methodological support for the standardization of traditional Chinese medicine (TCM) syndrome differentiation methods.

## 1. Introduction

Type 2 diabetes mellitus (T2-DM) is a chronic metabolic disease, causing significant increases in morbidity and mortality [1]. The global prevalence of diabetes has risen in adults from 4.7% in 1980 to 12.8% in 2018 [2]. The prevalence of type 2 diabetes in China is as high as 10.4%, showing an upward trend [3, 4]. Traditional Chinese medicine plays a more and more important role in the differential diagnosis and treatment of T2-DM [5]. Traditional Chinese medicine (TCM) is characterized by syndrome differentiation and treatment, which has been valuable to individualized clinical diagnosis and treatment. However, it is difficult to provide objective syndrome diagnosis by experiences. Also, previous clinical studies are not enough to reflect the characteristics of TCM. Therefore, it is crucial to study the objective standards for type 2 diabetes syndrome.

T2-DM is characterized by polydipsia, polyuria, and emaciation. Stomach heat flourishing (SHF) syndrome and Qi-Yin deficiency (QYD) syndrome are typical syndromes of T2-DM in clinical research of traditional Chinese medicine. In the early stage, swift digestion with rapid hungering and polydipsia is the outstanding characteristic of QYD syndrome [6]. With the aggravation of stomach heat consumption and yin injury, the symptoms of polydipsia, polyuria, and emaciation appear one after another. Stomach heat injures the kidney, resulting in kidney qi deficiency and kidney yin deficiency. Deficiency of kidney qi has no right to make urine clear and long, and kidney yin deficiency leads to yang hyperactivity, deficiency fire inflammation, that is, dizziness and tinnitus, insomnia, weakness of the waist and limbs, hot flashes, night sweats, and other yin deficiency syndromes, yin damage and yang deficiency, kidney yang deficiency and impotence, edema, and other symptoms. Deficiency of qi, deficiency of yin, and deficiency of yang can lead to the obstruction of blood flow and blood stasis, and blood stasis can cause many complications. In short, stomach heat is the key link in the pathogenesis of diabetes, and a variety of causes cause stomach heat, stomach heat injury yin, and gas consumption caused by both qi and yin injuries [7]. The evolution of T2-DM can be summarized as the beginning of the hyperactivity of stomach heat, followed by the injury of QYD syndrome. SHF syndrome is excess in superficiality, while QYD syndrome is the syndrome of deficiency in origin. Therefore, it is more significant to explore these two syndrome types in clinics.

Furthermore, there are growing statistical models and data mining methods that have been used in medical research [8–10]. In recent years, a variety of data analysis methods had also been used in the quantitative and objective diagnosis of TCM syndrome [11, 12]. Particularly, various researchers utilize the data mining method to extract the core attribute indicators of syndromes of T2-DM through the epidemiological investigation of clinical routine detection indicators of T2-DM. They formed a clear and instinctive judgment mode of the indicators made up for the inadequacy of traditional statistical methods [13, 14].

Our previous study found that the effective combination of clinical symptoms is helpful in the diagnosis of kidney yang deficiency syndrome and kidney yin deficiency syndrome. And the specific mixture of symptoms can mirror the situation of the patients with kidney deficiency [15]. Therefore, it is not only necessary but also possible to establish a syndrome diagnosis model constructed on data through the reasonable fusion of multiple data analysis methods [16–18]. Consequently, on the basis of a large number of clinical samples, combined with a variety of methods, the typical syndrome characteristics and effective index combination of T2-DM patients were analyzed, and the diagnosis model of two typical syndromes of T2-DM patients was established. At present, we established a diagnosis model of syndromes of T2-DM, explored symptoms, pulse and tongue signs, and laboratory indexes related to SHF syndrome and QYD syndrome by using the data mining methods, and compared the diagnostic power of three classification algorithms.

## 2. Materials and Methods

### 2.1. Data Source

From September 2013 to June 2017, 554 patients with type 2 diabetes were selected from the Department of Endocrinology, Chu Hsien-I Memorial Hospital (Metabolic Diseases Hospital) of Tianjin Medical University. All patients provided informed consent. The patients met the inclusion criteria and were differentiated by two associate chief physicians in traditional Chinese medicine.

### 2.2. Diagnostic Criteria for T2-DM

According to the “Guidelines for Prevention and Treatment of Type 2 Diabetes in China” (2017 Edition), the World Health Organization (WHO) (1999) diagnostic criteria for diabetes that are currently adopted in China, the epidemiological survey adopts fasting blood glucose 2 hPG or 75 g blood glucose after OGTT [4]. The conditions were as follows: (1) those with typical diabetes symptoms, such as polyuria, polyphagia, excessive drinking, and unexplained weight loss; plasma glucose level ≥11.1 mmol/L (200 mg/dL); (2) fasting plasma glucose (FPG) ≥7.0 mmol/L; (3) 2 h plasma glucose ≥11.1 mmol/L (200 mg/dL) using 75 g OGTT. If one of the above three conditions was met, the patient can be included, and the diagnosis can be confirmed by repeated tests.

### 2.3. TCM Diagnostic Criteria for T2-DM

The criteria of TCM diagnosis and syndrome differentiation of T2-DM are based on the terms of clinical diagnosis and treatment of TCM syndrome [19], guideline for clinical research of new drugs of TCM [20], diagnostics of TCM [21, 22], and internal medicine of TCM [23]. SHF syndrome includes dry mouth, dry throat, thirst, excessive drinking, frequent urination, constipation of stool, polyphagia, vulnerability to starvation, obvious weight loss, yellow fur, and smooth and slippery pulse. Symptoms such as polyphagia, vulnerability to starvation, emaciation, yellow fur, and smooth and slippery pulse can be diagnosed as indications of stomach heat flourishing syndrome. When there are three or more of the above symptoms identified, accompanied by reddish tongue with yellowish fur, slippery and rapid pulse can be diagnosed. QYD syndromes include dry mouth, dry throat, tired spirit, thirsty for drinking, poor appetite, spontaneous perspiration, thin body, reddish tongue, less moss, and weak pulse. When there are three or more of the above symptoms identified, accompanied by reddish tongue, weak pulse can be diagnosed.

### 2.4. Inclusion Criteria

The inclusion criteria were as follows: (1) patients aged from 18 to 70 were able to complete the questionnaire survey; (2) patients consistent with the diagnostic criteria of T2-DM developed by the WHO in 1999 and diagnosed as T2-DM at the time of the first diagnosis; (3) all patients had clear consciousness, had normal intelligence, and could accurately understand and answer the questions; (4) all patients signed informed consent; (5) all patients volunteered to participate in the investigation.

### 2.5. Exclusion Criteria

(1) Patients with type 1 diabetes or other diseases that cause elevated blood glucose, such as gestational diabetes, drug-induced diabetes, and severe liver disease caused by diabetes, stress hyperglycemia, increased glucocorticoids, and severe acute complications of diabetes; (2) patients with diabetic nephropathy stage IV or V and diabetic foot; systolic blood pressure >160 mmHg or diastolic blood pressure >100 mmHg after uncontrolled or controlled blood pressure; (3) patients with complications such as severe heart, lung, liver, acute, and chronic glomerular diseases, renal failure, acute and severe cardiovascular and cerebrovascular diseases, or with other serious primary diseases such as thyroid diseases (onset time <1 month); (4) women who are pregnant or lactating; (5) allergic constitution; (6) psychotic patient; (7) patients suffering from acute metabolic disorders such as trauma, surgery, hyperosmolar coma, and diabetic ketoacidosis in the last month.

### 2.6. Clinical Observation and Test Indexes

From the perspective of TCM and Western medicine, 58 symptoms and signs, 14 tongue signs, and 6 pulse signs were extracted by analyzing the literature of T2-DM in China National Knowledge Infrastructure (CNKI) and PubMed, and each patient was examined clinically. The general information of each patient included gender, nationality, marital status, age, occupation, education, past medical history, family history, height, weight, and blood pressure. The following laboratory indexes were investigated: fasting plasma glucose (FPG), 2-hour postprandial blood glucose, glycosylated hemoglobin A1c (HbA1C), oral glucose tolerance test (OGTT), total cholesterol (TC), triglyceride (TG), low-density lipoprotein (LDL), high-density lipoprotein (HDL), blood urea nitrogen (BUN), creatinine (CR), urinary glucose (UG), and urinary protein (UP).

### 2.7. Questionnaire Quality Control

1. Before the clinical and epidemiological investigation, under the guidance of physicians, the research manual of clinical investigation was carefully read by the investigators. As unified training was conducted and the analysis scheme was strictly implemented by an analyst, a measurement bias was reduced; (2) at least 2 clinical investigators shall be assigned to coordinate and supervise the work, and the case data shall be checked and improved regularly; (3) the questionnaire of T2-DM syndrome epidemiological information was uniformly used.

### 2.8. Data Management and Statistical Analysis

EpiData 3.1 is software used for the data management. The data were arranged in a column-wise format with each subject given a sequence identifier. Following the principle of independent input of two people, the questionnaire data were keyed by two people. In this study, continuous data with normal distribution were expressed as mean ± standard deviation (SD), while continuous data with no normal distribution were expressed as median (lower quartile, upper quartile). Data were expressed as a number and a percentage for categorical variables. If continuous data met the normal distribution and homogeneity of variance, the comparison of continuous variables between the two groups was performed by unpaired *t*-test; if continuous data did not fulfill the normal distribution or homogeneity of variance, the comparison of continuous variables between the two groups was performed via Wilcoxon rank-sum test. The comparison of categorical variables between the two groups was assessed by chi-square test or Fisher's exact test.

The method of logistic regression analysis in combination with quick, unbiased, efficient, statistical tree (QUEST) algorithm analysis was used in the study. 90 variables with multivariate were analyzed to compare the differences between SHF syndrome and QYD syndrome. These 90 variables were defined as independent variables while syndrome as a dependent variable. They were examined in a multivariate model by using forward stepwise maximum likelihood logistic regression to identify the symptoms (*α* = 0.05). Odds ratios (ORs) were estimated by multivariate logistic regression analysis. As shown in Table 1, the 90 variables were collected, and a complete clinical questionnaire of the TCM symptom set was constructed. All reported *P* values were those of two-sided tests. The statistical significance was set at *P* < 0.05.

The statistical algorithm that selected variables and quick, unbiased, efficient, statistical tree (QUEST) and CHAID algorithm analysis were used to develop the decision tree models. QUEST decision tree was a nonparametric procedure that made no assumptions of the underlying data. This algorithm determined how categorical independent variables can be combined without bias to predict a binary outcome based on the “if-then” logic and to build accurate binary trees quickly and efficiently. T2-DM syndrome was considered as a dependent variable, and 90 biological parameters were independent variables. However, we set “Parent Node” 100 and “Child Node” 50, allowing the tree model to grow sufficiently. Data were analyzed by using statistical software of SPSS version 25.0 for the logistic regression and decision tree model.

The *K*-nearest neighbor (KNN) method is an algorithm for classifying variables regarding the closest training data in the feature space. KNN is an instance-based learning method, which is one of the simplest algorithms among data mining methods. This method considers the nearest neighbors to each object and decides to dedicate the object to classes [24, 25]. In this paper, 10-fold cross-validation method was employed; that is, the dataset was divided into 10 parts, of which nine were taken in turn as the training set, the other was taken as the test set, and the average value of the results was used as the evaluation value of the algorithm performance.

## 3. Results

### 3.1. Sociodemographic Characteristics between SHF Syndrome and QYD Syndrome

In the 554 cases under investigation, 261 (47.1%) cases were diagnosed as SHF syndrome, while 293 (52.9%) cases were diagnosed as QYD syndrome by means of T2-DM syndrome differentiation criteria used by clinical experts in TCM. As shown from Table 1, among the 261 cases of SHF syndrome, 162 (62.1%) patients were male, and 99 (37.9%) were female, age *M* (*Q*_1_, *Q*_3_): 56.0 (48.0, 61.0). Among 293 cases with QYD syndrome, 141 (48.1%) patients were male, and 152 (51.9%) were female, age *M* (*Q*_1_, *Q*_3_): 57.7 (51.0, 66.0). Compared with QYD syndrome, lower proportions of SHF syndrome were females (37.9% versus 51.9%, *P*=0.001), the proportions of SHF syndrome were elder patients (27.2% versus 39.6%, *P*=0.003), lower proportions of SHF syndrome were with higher education (11.5% versus 6.9%, *P*=0.092), the proportions of SHF syndrome were white-collar employees (85.4% versus 85.7%, *P*=0.940), higher proportions of SHF syndrome were Han ethnics (98.1% versus 99.0%, *P*=0.602), higher proportions of SHF syndrome were married (86.2% versus 79.5%, *P*=0.038), lower proportions of SHF syndrome were with the past medical history (35.6% versus 29.0%, *P*=0.096), and proportions of SHF syndrome were with family history (50.6% versus 49.1%, *P*=0.737).

### 3.2. Multivariate Logistic Regression Analysis of Relevant Symptoms in Patients with the SHF Syndrome and QYD Syndrome

As shown from Table 2, logistic regression analysis showed that odor in the mouth, polyphagia, vulnerable to starvation, burning sensation in the stomach, slippery and replete pulse, OGTT, and hemoglobin A1C were relevant symptoms for the SHF syndrome. On the contrary, the symptoms, such as fatigue, limb weakness, weak pulse, and pink tongue were related with the QYD syndrome. The most significant symptoms of the differences between SHF syndrome and QYD syndrome were odor in the mouth, polyphagia, vulnerable to starvation, burning sensation in the stomach, slippery and replete pulse, OGTT, hemoglobin A1C, fatigue, limb weakness, weak pulse, and pink tongue (*P* < 0.05). As shown in Table 3, it was the result based on 554 cases of patients with symptoms. They were generated by the logistic regression model, which showed that 497 patients were classified accurately. The diagnostic accuracy was 89.7%. The sensitivity was 89.3%. The specificity was 90.1%.

### 3.3. QUEST Algorithm of Decision Tree Analysis: Establishment of the Identification Model on T2-DM Syndrome and Validation

The identification models of T2-DM syndrome were constructed by the QUEST decision tree, one of the algorithms of decision tree analysis. T2-DM syndrome was considered as a dependent variable, whereas 11 attributes of TCM (including 6 symptoms, 2 pulse signs, 1 tongue sign, and 2 laboratory indexes) were labeled as independent variables. “Parent Node” 100 and “Child Node” 50 were set up which allowed the tree model to develop sufficiently. The decision tree algorithms divide data into statistically significant subgroups, which are exclusive and detailed to both parties [24]. In order to increase the operability of clinical application, the number of branches of the decision tree is limited to 4. As shown in Figure 1, in this model, the tree analysis showed the 2-level QUEST decision tree with a total of 7 nodes, of which 4 were terminal nodes. Three major predictors of symptoms which reached significance and were included in this model were demonstrated as slippery and replete pulse, polyphagia, and weak pulse. The other 57 symptoms, 14 tongue signs, 4 pulse signs, and 12 laboratory indexes were not significant in the model. As shown in Table 3, the diagnostic model used to differentiate these two types of T2-DM among 554 cases had an overall accurate diagnostic rate of 85.2%, with the sensitivity of 78.2% and specificity of 91.5%, respectively.

The first level of the QUEST decision tree was split into two initial branches in terms of the first level on slippery and replete pulse. The symptom of slippery and replete pulse was the best symptom to identify SHF syndrome, and the classification accuracy of SHF syndrome was at 89.1%. On the contrary, 82.5% of patients with no slippery and replete pulse were identified as QYD syndrome. As seen in the second level of the QUEST decision tree, weak pulse was the next best predictor variable for cases. The classification accuracy of QYD syndrome was 99.0% for patients with weak pulse. At the same time, accurate diagnostic rate of SHF syndrome for patients with polyphagia was 100%.

### 3.4. Results of CHAID Algorithm of Decision Tree Analysis: External Validation Mode for T2-DM Syndrome

With the CHAID decision tree method, an external validation mode for SHF syndrome and QYD syndrome for 554 T2-DM patients was made up of three biological parameters. As shown in Figure 2, the number of nodes in this mode was 9, and the number of terminal nodes was 5. The mode was much more complex for these 3 parameters formed 8 identification paths for SHF syndrome and QYD syndrome. Smooth and replete pulse was the best predictor of SHF syndrome and QYD syndrome. The second-grade variable quantity was polyphagia and weak pulse, and the third-grade variable was polyphagia. As shown in Table 3, the result of 10-fold cross-validation was shown for SHF syndrome and QYD syndrome in the external validation mode with the sensitivity of 78.2% and specificity of 91.5%, respectively. The percentage of correct prediction was 85.2%.

### 3.5. Results of the *K*-Nearest Neighbor Method: Identification Model on T2-DM Syndrome

As shown from Table 3, the classification model used to differentiate the two types of T2-DM among 554 cases had an overall accurate classified rate of 88.3%, with the sensitivity of 84.7% and specificity of 91.5%, respectively. Three major predictors of symptoms were the nearest neighbors to the two types of T2-DM in the model which were demonstrated as slippery and replete pulse, polyphagia, and weak pulse.

### 3.6. Comparison of the Area under the ROC Curve of Three Classification Methods

The sensitivity, specificity, and AUC of three classification methods have been demonstrated in Table 3. Area under the ROC curve (AUC) computes the entire two-dimensional area under the whole ROC curve. According to the finding, AUC dedicated to logistic regression is bigger among the methods. Apart from classification sensitivity, specificity, and AUC, the receiver operating characteristic (ROC) is shown for each approach in Figure 3. A larger area under the curve (AUC) is usually better. According to the demonstrated ROCs, the logistic regression has a better area under the curve in comparison with the decision tree and *K*-nearest neighbor method.

## 4. Discussion

T2-DM is a common and frequent disease of endocrine metabolic disease, belonging to the category of Xiao Ke disease in TCM. “*Synopsis of the Golden Chamber*” written by Zhang Zhongjing in the Eastern Han Dynasty is the earliest classical book of traditional Chinese medicine. It points out that “fighting between the hard and the weak” means that the stool is hard, and frequent urination is the key point of pathogenesis. It reflects that excessive lung and stomach heat leads to excessive drinking, and swift digestion with rapid hungering is excess in superficiality, while Qi-Yin deficiency due to unfavorable gasification is deficiency in origin. Intake of water cannot be retained in the body; it will become body fluid and be excreted from the kidneys. The earliest syndrome types of T2-DM can be divided into two types: SHF syndrome and QYD syndrome. SHF syndrome is excess in superficiality, while QYD syndrome is the syndrome of deficiency in origin. Therefore, it is necessary to establish an identification model of typical syndromes of T2-DM, SHF syndrome and QYD syndrome, by using the data mining methods.

Several studies have investigated different data mining methods to identify Chinese medicine syndrome of different diseases such as metabolic syndrome, coronary heart disease, IgA nephropathy, chronic hepatitis B, and acute exacerbation of chronic obstructive pulmonary disease [9, 11, 12, 26, 27]. In the present study, the clinical manifestations of 554 cases with T2-DM syndrome are complicated, which is the observation basis of TCM syndrome differentiation treatment. In the clinical investigation, SHF syndrome and QYD syndrome are the two main syndrome types of T2-DM. The diagnostic models of SHF syndrome and QYD syndrome with T2-DM in patients were established and compared by using logistic regression, decision tree, and *K*-nearest neighbor method. Logistic regression analysis showed that odor in the mouth, polyphagia, vulnerable to starvation, burning sensation in the stomach, slippery and replete pulse, OGTT, hemoglobin A1C, fatigue, limb weakness, weak pulse, and pink tongue were the most significant symptoms of the differences between SHF syndrome and QYD syndrome (*P* < 0.05). However, the decision tree and *K*-nearest neighbor method are more consistent in dealing with the relationship among only three symptoms selected: slippery and replete pulse, polyphagia, and weak pulse. As shown in Figures 1 and 2, there were obvious differences in the occurrence rates of these three symptoms in patients with SHF syndrome and QYD syndrome. Therefore, it was reasonable that these three symptoms, such as slippery and replete pulse, polyphagia, and weak pulse, were selected and placed in the decision tree model and *K*-nearest neighbor model. However, the occurrence rates of six symptoms, odor in the mouth, vulnerability to starvation, burning sensation in the stomach, fatigue, OGTT, and hemoglobin A1C, were not the nearest to the two syndromes, so they were excluded from the decision tree model. The combination of logistic regression and decision tree has also been proved to be effective in modern medical diagnosis [28, 29]. In this study, the diagnostic accuracy of the logistic regression model and decision tree model for the two syndromes was basically consistent (logistic regression model was 87.7%, and decision tree model was 80.3%). However, 11 indicators, such as odor in the mouth, polyphagia, vulnerability to starvation, burning sensation in the stomach, slippery and replete pulse, OGTT, hemoglobin A1C, fatigue, limb weakness, weak pulse, and pink tongue were analyzed by using the logistic regression model, while only 3 indicators, such as slippery and replete pulse, polyphagia, and weak pulse were analyzed by using the decision tree model. In addition, the decision tree is a nonparametric method [30], and the representation of its model is easier to understand and more practical, which is also convenient for the actual operation of clinical syndrome diagnosis.

LR, DT, and KNN suggest that symptoms and pulse diagnosis are of great significance in the differentiation of type 2 diabetes. At the same time, slippery and replete pulse, polyphagia, and weak pulse in different diagnostic models have a good effect on the differential diagnosis of SHF syndrome and QYD syndrome, which is consistent with the experience of TCM syndrome differentiation. The study also showed that the combination of laboratory examination indexes and some specific symptoms of TCM in patients has the value of syndrome differentiation [31]. The study also showed that QYD syndrome was associated with hemoglobin A1C [32]. Therefore, it is a new idea to explore objective research studies on the syndrome of some modern laboratory indicators and understand the combination relationship between symptoms of TCM and laboratory indicators. Applying data mining methods to identify T2-DM syndrome diagnosis may assist practitioners to enhance the quality of their clinical decisions.

As shown from the results, KNN has a lower area under the curve in comparison with DT and LR. The structure of the data may lead to the difference. In addition, KNN is a nonparametric learning method, which cannot reflect the influence of each independent variable on the dependent variable. Consequently, DT is fitter to the data. As everyone knows, the fundamental difference between DT models and both LR and KNN is that DT models learn step functions. Therefore, identification models of T2-DM syndrome depend on the relationship of variables. DT shows better identification than LR when nonlinear correlation occurs between independent and dependent variables. When there is a step function correlation between the variables, DT model is more suitable for the classification of T2-DM syndrome. So, DT has obvious advantages in expressing the rules of syndrome differentiation, which is suitable for the main technical method of TCM syndrome diagnosis.

In conclusion, the model between SHF syndrome and QYD syndrome in patients with T2-DM was initially constructed in the study in order to provide new methods and new ideas for T2-DM patients to diagnose and treat SHF and QYD syndromes from the perspective of traditional Chinese medicine. The results show that the reasonable combination of some laboratory indexes and TCM syndromes has certain dialectical significance. This suggests that the combination of multiple statistical analysis models is a feasible method to improve the objectivity of syndrome diagnosis. In the future, it is necessary to test the reliability of the model in new clinical patients and carry out the comprehensive investigation of large clinical samples and multiple syndromes to further improve the diagnostic accuracy and stability of the model and comprehensively establish a diagnostic model containing multiple syndromes. Moreover, the relationship between qualitative and quantitative indexes with syndrome differentiation and their biological basis was to be studied.

## Figures and Tables

**Figure 1:** QUEST algorithm of decision tree analysis of T2-DM syndrome.

**Figure 2:** CHAID algorithm of decision tree analysis of T2-DM syndrome.

**Figure 3:** Comparison of the area under the ROC curve of three classification methods.

**Table 1:** Comparison of sociodemographic characteristics between the SHF syndrome and QYD syndrome.

Total	T2-DM syndrome		Statistics value	*P* value
	SHF syndrome (*n* = 261)	QYD syndrome (*n* = 293)		
Gender	*N* (%)	*N* (%)		
Male	162 (62.1)	141 (48.1)^*∗*^	10.834	0.001
Female	99 (37.9)	152 (51.9)		
Age (years)				
<40	36 (13.8)	24 (8.2)^*∗*^	11.422	0.003
40–60	154 (59.0)	153 (52.2)		
>60	71 (27.2)	116 (39.6)		
*M* (*Q*_1_, *Q*_3_)	56.0 (48.0, 61.0)	57.7 (51.0, 66.0)^*∗*^	3.558	<0.001
Education (years)				
6	28 (10.7)	42 (14.3)	4.774	0.092
12	203 (77.8)	231 (78.8)		
≥13	30 (11.5)	20 (6.9)		
Occupation				
White collar	223 (85.4)	251 (85.7)	0.006	0.940
Blue collar	38 (14.6)	42 (14.3)		
Ethnic				
Han nationality	256 (98.1)	290 (99.0)	0.272	0.602
Others	5 (1.9)	3 (1.0)		
Marital status				
Married	225 (86.2)	233 (79.5)^*∗*^	4.306	0.038
Unmarried	36 (13.8)	60 (20.5)		
Past medical history				
Yes	93 (35.6)	85 (29.0)	2.776	0.096
None	168 (64.4)	208 (71.0)		
Family history				
Yes	132 (50.6)	144 (49.1)	0.113	0.737
None	129 (49.4)	149 (50.9)		

^∗^Female patients with T2-DM are more prone to develop QYD syndrome, while male patients with T2-DM are more likely to develop SHF syndrome. Elderly patients with T2-DM are more prone to develop QYD syndrome, while young and middle-aged diabetic patients are more likely to develop SHF syndrome. The ratio of SHF syndrome of married patients with T2-DM is higher than that of QYD syndrome.

**Table 2:** Logistic regression of symptoms associated with SHF syndrome and QYD syndrome.

Variable	*B*	SE	Wald	df	*P*	Exp (*B*)	OR (95% CI)
Odor in the mouth	0.688	0.322	4.557	1	0.033	1.989	(1.058, 3.741)
Fatigue	−0.787	0.395	3.969	1	0.046	0.455	(0.210, 0.987)
Limb weakness	−0.907	0.386	5.527	1	0.019	0.404	(0.189, 0.860)
Polyphagia	1.734	0.357	23.549	1	<0.001	5.661	(2.811, 11.401)
Vulnerable to starvation	0.666	0.333	4.002	1	0.045	1.947	(1.014, 3.739)
Burning sensation in the stomach	1.527	0.421	13.163	1	<0.001	4.606	(2.018 10.511)
Slippery and replete pulse	4.021	0.382	110.545	1	<0.001	55.752	(26.347, 117.974)
Weak pulse	−3.682	0.777	22.438	1	<0.001	0.025	(0.005, 0.115)
Pink tongue	−0.860	0.360	5.706	1	0.017	0.423	(0.209, 0.857)
Oral glucose tolerance test (OGTT)	0.178	0.068	6.922	1	0.009	1.194	(1.046, 1.363)
Hemoglobin A1C (HbAlc)	0.152	0.062	5.927	1	0.015	1.164	(1.030, 1.316)

**Table 3:** Results of three classification methods for 554 cases with T2-DM syndrome.

Method	T2-DM syndrome	TN	FP	Sensitivity (%)	Specificity (%)	Accuracy (%)	AUC
		FN	TP				
LR	SHF syndrome	233	28	89.3	90.1	89.7	0.953
	QYD syndrome	29	264				

QUEST algorithm of DT	SHF syndrome	204	57	78.2	91.5	85.2	0.931
	QYD syndrome	25	268				

CHAID algorithm of DT	SHF syndrome	204	57	78.2	91.5	85.2	0.931
	QYD syndrome	25	268				

KNN	SHF syndrome	211	40	84.7	91.5	88.3	0.887
	QYD syndrome	15	278				

Sensitivity = TP/(TP + FN); specificity = TN/(TN + FP); accuracy = (TP + TN)/(TP + FN + TN + FP).

## Data Availability

The original data are not available publicly.

## Abbreviations

AUC: Area under the ROC curve
BUN: Blood urea nitrogen
CHAID: Chi-squared automatic interaction detector
CNKI: China National Knowledge Infrastructure
DM: Diabetes mellitus
DT: Decision tree
FPG: Fasting plasma glucose
HbA1C: Hemoglobin A1C
HDL: High-density lipoprotein
KNN: *K*-nearest neighbor
LDL: Low-density lipoprotein
LR: Logistic regression
OGTT: Oral glucose tolerance test
QUEST: Quick, unbiased, efficient, statistical tree
QYD: Qi-Yin deficiency syndrome
ROC: Receiver operating characteristic
SHF: Stomach heat flourishing syndrome
TC: Total cholesterol
TCM: Traditional Chinese medicine
TG: Triglyceride
T2-DM: Type 2 diabetes mellitus
UG: Urinary glucose
UP: Urinary protein
2hPG: 2-hour postprandial glucose.
